# Adoption of Dexmedetomidine in Different Doses at Different Timing in Perioperative Patients

This article has been retracted.

**DOI:** 10.1155/2022/4008941

**Published:** 2022-07-15

**Authors:** Jing Xie, Shiqiang Feng, Zhenhua Qu

**Affiliations:** Department of Anesthesiology, Xingtai People's Hospital, Xingtai, Hebei, China

## Abstract

Dexmedetomidine (Dex) is an alpha-2 agonist used for sedation during various procedures. Dex activates 2-adrenoceptors, and causes the decrease of sympathetic tone, with attenuation of the neuroendocrine and hemodynamic responses to anesthesia and surgery; it reduces anesthetic and opioid requirements; and causes sedation and analgesia. Objective: it was to compare the perioperative effects of different doses of Dex at different timing in patients using Dex during the perioperative period adopting a medical data classification algorithm based on optimized semi-supervised collaborative training (Tri-training). Methods: 495 patients requiring surgical treatment in Xingtai People's Hospital were randomly selected as the study subjects. The patients were divided into group A (used before induction), group B (used during induction), and group C (used after induction) according to different induction timing, with 165 cases in each group. Then, groups A, B, and C were divided into groups A1, B1, and C1 (0.4 *μ*g/(kg·h) rate), groups A2, B2, and C2 (0.6 *μ*g/(kg·h) rate), and groups A3, B3, and C3 (0.8 *μ*g/(kg·h) rate) according to the dose used, with 55 cases in each group. Intraoperative anesthesia and postoperative adverse reactions were compared among the 9 groups. Results: the similarity between the Tri-training algorithm optimized by Naive Bayes (NB) classification algorithm and the actual classification (93.49%) was clearly higher than that by decision tree (DT) and K-nearest neighbor (kNN) classification algorithm (76.21%, 74.31%); heart rate (HR), systolic blood pressure (SBP), and diastolic blood pressure (DBP) values decreased obviously after Dex used in groups B1, C1, B2, C2, B3, and C3 (*P <0.05*), but did not change significantly in groups A1, A2, and A3 (*P >0.05*); the proportion of patients with satisfactory Ramsay score in group A3 was distinctly superior than that in groups A1, A2, B1, B2, B3, C1, C2, and C3 (*P <0.05*); the incidence of adverse reactions in group A3 was significantly inferior than that in groups A1, A2, B1, B2, B3, C1, C2, and C3 (*P <0.05*). Conclusion: the optimization effect of NB classification algorithm was the best, and the injection of Dex at the injection rate of 0.8 *μ*g/(kg·h) before induction of anesthesia could apparently improve the fluctuation of HR, SBP, and DBP during perioperative period, and effectively reduce the occurrence of adverse reactions in patients, with better sedative effect on patients.

## 1. Introduction

Anesthesia is one of the necessary operation steps in the surgical treatment of most diseases in clinical practice. Clinical time shows that more sedative drugs are often required to strengthen and maintain the anesthetic effect during surgery, thereby reducing the patient's pain during surgery. However, there are some risks in the use of anesthetic drugs. Through the summary of previous clinical application experience, inappropriate use of anesthetics will lead to certain damage to the central nervous function of patients, resulting in a series of complications, such as increased blood pressure, language impairment, cognitive impairment. In addition, some studies have proposed that the patient's mood before anesthesia has a certain impact on the anesthetic effect, therefore, mood induction during the whole process of anesthesia is relatively important [1].

Dexmedetomidine (Dex) is a highly selective *α*2-adrenoceptor agonist that is soluble [2]. In recent years, the clinical application of Dex has been widely studied. Studies have shown that Dex has a rapid onset of action during sedation, little impairment of neurological function, and does not produce respiratory depression [3, 4]. Therefore, the clinical application of Dex has received more attention from experts. Dex has been used in the perioperative period of gynecological malignancy surgery [5], laparoscopic hepatobiliary surgery [6], and thyroid surgery [7]. It has been proposed that preoperative administration of 0.8 *μ*g/(kg · h) Dex is superior to 0.4 *μ*g/(kg · h) [8]. It has also been presented that the use of Dex during induction of anesthesia is more effective than before and after induction [9]. However, there is no clinical study on when and at what dose Dex is best used in the perioperative period. In order to better play the intervention effect of Dex in the perioperative period and reduce the incidence of adverse reactions, it focuses on surgical patients with different diseases to explore the optimal timing and optimal dose of Dex.

The study subjects were selected nationwide. Then, it is necessary to consider the classification and collation of big data (BD) in research, especially the rapid development of information technology nowadays, the type and scale of medical data have been rapidly grown [10]. The method using artificial intelligence (AI) was put forward to get more reasonable classification and collation of medical data [11]. Traditional AI algorithms are often performed under supervised learning, but their application on “labelling” data information is very difficult and requires a lot of manpower and material resources to support [12]. Therefore, the data classification function of supervised learning is limited. In order to better classify and sort medical data, some experts point out a semi-supervised collaborative training (Tri-training) algorithm [13]. Semi supervised learning is one of the prominent ways to address the problem of limited labeled samples by learning from both labeled and unlabeled samples without human intervention. In semi supervised learning, an effective paradigm is referred to as disagreement-based semi supervised learning, where multiple base learners are trained and they learn from each other collaboratively to improve the performance by exploiting the disagreement among them. This algorithm has been applied in the classification of coronary heart disease (CHD), and has achieved good application results. However, it has been concluded that for unlabelled classification data, the accuracy of Tri-training algorithm for data classification is greatly limited and further optimization is needed [14].

To obtain the optimal timing and dose of Dex and to ensure a more representative discussion, the optimized Tri-training medical BD classification algorithm was adopted to explore the perioperative anesthesia of patients with Dex in 100 tertiary hospitals nationwide, and compare the effects of different doses of Dex at different time during perioperative period. It was to improve the clinical sedative effect in the process of surgical treatment, and to improve the postoperative rehabilitation and prognosis of patients.

## 2. Materials and Methods

### 2.1. Study Subjects and Grouping

A total of 495 patients requiring surgical treatment from March 2021 to March 2022 in Xingtai People's Hospital were randomly selected as the study subjects. After statistical classification, there were 284 male patients and 211 female patients, with age range of 20~60 years, mean age of (41.39 ± 9.12) years, weight of 45~80 kg, and mean weight of (50.45 ± 14.05) kg. There were 156 patients who underwent gynecological malignant tumor surgery, 206 patients who underwent laparoscopic hepatobiliary surgery, and 133 patients who underwent subtotal thyroidectomy under general anesthesia. According to the induction timing of Dex, the patients were divided into group A (used before induction), group B (used during induction), and group C (used after induction), with 165 cases in each group. Then, groups A, B, and C were divided into groups A1, A2, A3; B1, B2, B3; C1, C2, and C3, respectively, according to different doses used, with 55 patients in each group. Patients in groups A1, B1, and C1 were treated with 0.4 *μ*g/(kg·h) intravenous drip, patients in groups A2, B2, and C2 were treated with 0.6 *μ*g/(kg·h) intravenous drip, and patients in groups A3, B3, and C3 were treated with 0.8 *μ*g/(kg·h) intravenous drip. Intraoperative anesthesia and postoperative adverse reactions were compared among the 9 groups. The experiment was approved by the relevant medical ethics committee.

Inclusion criteria: patients aged over 18 years old; patients who volunteered to participate in this experiment and signed the informed consent; patients with clear mental consciousness; all patients were induced with Dex.

Exclusion criteria: patients allergic to anesthetic drugs; patients with severe dysfunction of heart, liver, kidney, lung, and other organs and severe metabolic diseases; patients suffering from mental illness; patients who take psychotropic drugs for a long time; patients who abuse anesthetic and analgesic drugs; patients who take antihypertensive drugs; patients who do not undergo complete surgery.

### 2.2. Data Classification Based on tri-Training Algorithm

Tri-training algorithm is to train three base classifiers through supervised learning algorithm, combine them pairwise to classify unlabelled data, and expand and train the remaining classifiers, to improve the performance of base classifiers. Its main algorithm structure is shown in Figure 1.

The specific algorithm process is as follows.

It is assumed that the marked data set is *Q*, the unlabelled data set is *q*, *H* represents the base classifier and *L* represents the initial training set, and the following equation can be obtained.

(1) $$\begin{array}{c} H_{t}=Base\;classifier\left(Q\right) \end{array}$$

(2) $$\begin{array}{c} L_{t}=Base\;classifier\left(q\right) \end{array}$$

*t* represents the type of base classifier and training set, *t* ∈ [1, 2, 3]. All parameters are initialized to obtain $\left\{\begin{array}{c} w_{t}=0.5\\ L_{t}=0 \end{array}\right.$, and *w* means the upper limit of classification error rate. When *t* = [1, 2, 3], Equation (3) is obtained.

(3) $$\begin{array}{c} L_{t}\neq 0,w_{t}=Error \end{array}$$

(4) $$\begin{array}{c} L_{t}=\left|\frac{w_{t}}{w_{t-1}-w_{t}}+1\right| \end{array}$$

(5) $$\begin{array}{c} L\prime_{t}=\left|\frac{w_{t}L_{t}}{w_{t}}-1\right| \end{array}$$

After calculations, the final classifier *f*(*t*) can be obtained.

(6) $$\begin{array}{c} f\left(x\right)=\arg\underset{z=C}{\max}\int_{t:L_{t}\left(x\right)=z}1 \end{array}$$

Because the Tri-training algorithm adopts implicit setting, the accuracy of implicit confidence is lower than that of explicit confidence. It will be optimized in combination with class probability estimation. The class probability estimation algorithms of common classifiers include decision tree (DT) Decision trees use multiple algorithms to decide to split a node into two or more sub-nodes. The creation of sub-nodes increases the homogeneity of resultant sub-nodes [15], Naive Bayes (NB) It is a classification technique based on Bayes' Theorem with an assumption of independence among predictors. In simple terms, a Naive Bayes classifier assumes that the presence of a particular feature in a class is unrelated to the presence of any other feature [16], K-nearest neighbor (kNN) K Nearest Neighbor algorithm falls under the Supervised Learning category and is used for classification (most commonly) and regression. It is a versatile algorithm also used for imputing missing values and resampling datasets [17].

The DT classifies the data according to the tree structure, and uses the probability distribution on the leaf nodes to predict the classification of the data. The specific calculation is as below.

(7) $$\begin{array}{c} DT\left(C_{i}\left|x,m\right.\right)=\frac{\int_{j=1}^{N}\beta \in \left(C_{i},C_{j}\right)}{N}. \end{array}$$

*N* represents the total number of training samples in the leaf node; *m* represents leaf nodes; *C_i_* indicates the leaf node category; *C*_*j*_ represents the category of the sample *C*_*j*_.

NB is based on Bayes theorem and classifies data by analyzing the joint probability distribution of data input and output. n probability theory and statistics, Bayes' theorem (alternatively Bayes' law or Bayes' rule; recently Bayes–Price theorem, named after Thomas Bayes, describes the probability of an event, based on prior knowledge of conditions that might be related to the event. One of the many applications of Bayes' theorem is Bayesian inference, a particular approach to statistical inference. When applied, the probabilities involved in the theorem may have different probability interpretations. With Bayesian probability interpretation, the theorem expresses how a degree of belief, expressed as a probability, should rationally change to account for the availability of related evidence. Bayesian inference is fundamental to Bayesian statistics.

(8) $$\begin{array}{c} NB\left(C_{i}\left|x\right.\right)=NB\left(C_{i}\right)\int_{j=1}^{\dim}NB\left(A_{j},C_{i}\right) \end{array}$$

dim refers to the characteristic dimension of the target sample; *j* refers to order; *A* refers to characteristics; *NB*(*C*_*i*_) refers to the prior probability distribution of the sample; *NB*(*A*_*j*_, *C*_*i*_) means the conditional probability distribution.

*kNN* is a relatively simple and effective classification method, which selects *k* samples closest to the sample *x* for statistical classification of data.

(9) $$\begin{array}{c} kNN\left(C_{i}\left|x\right.\right)=k_{m}/k \end{array}$$

*k_m_* is the number of *C*_*i*_ of *k* samples.

(10) $$\begin{array}{c} k=2n+1\left(n\in 0,1,\cdots ,\infty \right) \end{array}$$

The structure diagram of the classification model of Tri-training algorithm after class probability estimation algorithm is as follows, which is mainly divided into two modules: training and testing (Figure 2).

The clinical data of 2,010 patients with CHD were selected as the test object to classify and sort out the types of CHD, test the optimization effect of the above three classification algorithms (DT, NB, kNN), and evaluate the similarity between the classification results and the actual situation.

(11) $$\begin{array}{c} \text{Similarity}=\left({\text{R}}_{\text{Algorithm}}/R_{\text{Reality}}\right)\times 100\% \end{array}$$

### 2.3. Anaesthetic Method

The patients in group A, group B, and group C were given the same anesthesia method (before surgery, fasting for 6 ~ 8 h, prohibition of drinking for 2 h) and monitored by routine monitoring of electrocardiogram (ECG), pulse, and oxygen saturation (SpO_2_). Afterwards, intravenous anesthesia was carried out using propofol (the initial plasma target concentration was 2.5 *μ*g/mL) and 3 *μ*g/kg of fentanyl. 0.15 mg/kg of atracurium was given when the patient's consciousness disappeared (drugs from Xuzhou Ryen Pharma Co., Ltd.). Patients in group A were injected with 0.4 *μ*g/kg, 0.6 *μ*g/kg, and 0.8 *μ*g/kg of Dex hydrochloride before induction of anesthesia; patients in group B were given during induction of anesthesia; and patients in group C were injected after induction. They were then sent to the anesthesia recovery room after the end of surgery for continued observation until recovery.

### 2.4. Observation Indexes

The heart rate (HR), systolic blood pressure (SBP), and diastolic blood pressure (DBP) of patients in each group were recorded before anesthesia, after anesthesia, during intubation, 5 minutes after intubation, and 30 minutes after intubation.

Sedation score (Ramsay) after extubation [18] (Table 1) and occurrence of perioperative adverse events (severe bradycardia, hypotension, hypertension, dry mouth, nausea, vomiting, etc.) were recorded. RAMSAY scale had been originally developed to be used only for sedated patients to monitor level of sedation. It divides a patient's level of sedation into six categories ranging from severe agitation to deep coma.

### 2.5. Statistical Methods

SPSS 23.0 calculation system was used for data analysis, and measurement data were expressed by *t*-test and ($\overset{¯}{\text{x}}$±s). Enumeration data were expressed by *χ*^2^ and percentage (%), and *P <0.05* indicated statistical significance.

## 3. Results and Discussion

### 3.1. Classification Accuracy of Algorithm

Through calculating the classification results and actual classification of disease types of 2,010 patients with CHD by DT, NB, and kNN classification algorithms, it was concluded that the similarity between Tri-training algorithm optimized by NB classification algorithm and actual classification (93.49%) was significantly higher than that by DT and kNN classification algorithms (76.21%, 74.31%) (Figure 3). The results suggested that the NB classification algorithm had the best optimization effect on the Tri-training algorithm. NB classification algorithm has been extensively studied at present. For example, Mansour et al. (2021) [19] used NB classification algorithm for coronavirus (COVID-19) prediction, and Wood et al. (2019) [20] applied it in the analysis of cancer data. The above findings revealed that NB classification algorithm had a good application effect in various fields. Moreover, Ngabo *et al.* (2021) [21] also utilized the above three algorithms for classification prediction of epidemic diseases and compared them, and the results also showed that NB had the best application effect in data classification. The conclusion was consistent with the results of this experiment, and also provided reasonable support for the results. On this basis, a subsequent exploration was conducted to analyze and evaluate the timing and dosage of Dex.

### 3.2. Comparison of General Data

495patients were divided into groups A1, A2, A3; B1, B2, B3; C1, C2, and C3 according to the timing and dose of application. The general clinical data (gender, age, weight, type of surgery) of the nine groups were statistically analyzed by classification algorithm, and the following results were obtained: (1) Gender distribution: 33, 34, 32, 28, 30, 32, 31, 32, and 31 male patients, respectively; 22, 21, 23, 27, 25, 23, 24, 22, and 24 female patients, respectively, in the nine groups. (2) Distribution of mean age: The mean age of the nine groups was (40.01 ± 10.19) years, (42.19 ± 8.22) years, (40.67 ± 9.01) years, (41.09 ± 8.82) years, (42.11 ± 9.05) years, (42.23 ± 9.22) years, (40.09 ± 8.74) years, (40.67 ± 9.42) years, and (41.94 ± 10.92) years, respectively. (3) Average weight distribution: The average weight of patients in the nine groups was (50.01 ± 13.05) kg, (51.12 ± 15.00) kg, (49.07 ± 16.05) kg, (50.22 ± 13.95) kg, (52.03 ± 15.02) kg, (50.11 ± 14.11) kg, (51.22 ± 13.95) kg, (50.29 ± 14.89) kg, and (52.98 ± 14.98) kg, respectively. (4) Distribution of surgical types: 34.56%, 36.36%, 32.72%, 34.56%, 34.56%, 34.56%, 34.56%, 34.56%, and 34.56% of the patients in the nine groups underwent gynecological malignant tumor surgery; 38.18%, 36.36%, 38.18%, 40.00%, 34.55%, 36.36%, 40.00%, 38.18%, and 36.36% of the patients underwent laparoscopic hepatobiliary surgery; and 27.27%, 27.27%, 29.09%, 25.45%, 30.91%, 29.09%, 25.45%, 27.27%, and 25.45% of the patients underwent subtotal thyroidectomy under general anesthesia. The comparison showed that there was no significant difference in the distribution of gender, age, weight, type of surgery among groups A1, A2, A3, B1, B2, B3, C1, C2, and C3 (*P* <0.05) (Figure 4).

### 3.3. Hemodynamic Comparison

The effects of groups A1, A2, A3, B1, B2, B3, C1, C2, and C3 on hemodynamics HR, SBP, and DBP were compared before anesthesia, after anesthesia, during intubation, 5 min after intubation, and 30 min after intubation.  Figure 5 indicated the injection volume of 0.4 *μ*g/(kg · h), the HR, SBP, and DBP results of patients in groups A1, B1, and C1 before anesthesia, after anesthesia, during extubation, 5 min after extubation, and 30 min after extubation. According to the results, there was no significant difference in HR, SBP, and DBP among the three groups before anesthesia (*P >0.05*), but the HR, SBP, and DB*P* values of patients in groups B1 and C1 after application of Dex decreased (*P <0.05*), while those of patients in group A1 were no obvious change (*P >0.05*), suggesting that the perioperative hemodynamic changes in group A1 were relatively stable.

Figure 6 showed the injection volume of 0.6 *μ*g/(kg · h), the results of HR, SBP and DBP of patients in groups A2, B2 and C2 before anesthesia, after anesthesia, during extubation, 5 min after extubation, and 30 min after extubation were compared.  Figure 7 showed the injection volume of 0.8 *μ*g/(kg · h), HR, SBP, and DBP results of patients in groups A3, B3, and C3 before anesthesia, after anesthesia, during extubation, 5 min after extubation, and 30 min after extubation. Through analysis, the change trend of HR, SBP, and DBP results in Figures 6 and 7 was consistent with Figure 5. In other words, the hemodynamic changes of patients in groups A1, A2, and A3 were less, and the values of HR, SBP, and DBP in different periods were more stable.

From the above results, Dex injection before induction of anesthesia could improve the changes in blood pressure and HR caused by anesthesia in patients. The purpose of induction of surgical anesthesia was to improve the depth of anesthesia and reduce the stress response caused by tracheal intubation or surgical stimulation (non-specific defense response caused by strong stimulation), improving the adverse hemodynamic fluctuation of patients [22]. Before anesthesia, patients often have decreased blood volume due to adverse emotions to surgical treatment, causing excessive changes in blood pressure and heart rate as well as reduced body tolerance. Li et al. (2019) [23] suggested that Dex injection before anesthesia could effectively relieve perioperative hemodynamics and protect myocardial cells in thoracic surgery. Elgebaly *et al*. (2020) [24] found that Dex was more effective before anesthesia.

The HR, SBP, and DBP of groups A1, A2, and A3 before anesthesia, after anesthesia, during intubation, 5 min after intubation, and 30 min after intubation were statistically compared. The results were given in Figure 8. The HR, SBP, and DB*P* values of group A3 were more stable than those of group A1 and A2 at different time points. The results showed that Dex had the best sedative effect when the injection dose was 0.8 *μ*g/(kg · h). Shamim et al. (2017) [25] proposed that Dex was more effective at an injection dose of 0.7 ~ 0.8 *μ*g/kg · h than at 0.4 ~ 0.6 *μ*g/kg · h at the same injection timing. It was also in line with the findings of Ramachandran et al. (2021) [26]. Therefore, before induction of anesthesia, 0.8 *μ*g/(kg · h) of Dex had the best sedative effect.

### 3.4. Comparison of Ramsay Score Results

Table 2 shows the distribution of Ramsay scores of patients in groups A1, A2, A3, B1, B2, B3, C1, C2, and C3. After calculation, the satisfaction of sedation effect of patients in groups A1, A2, A3, B1, B2, B3, C1, C2, and C3 was 90.91%, 89.09%, 96.36%, 87.27%, 87.27%, 90.91%, 89.09%, 89.09%, 85.45%, respectively. Through observation, the proportion of patients with satisfactory sedation in group A3 was significantly higher than that in groups A1, A2, B1, B2, B3, C1, C2, and C3 (*P <0.05*). Ramsay sedation score scale is an effective and reliable evaluation scale for sedation monitoring of invasive operation under deep sedation, which has been widely used in related clinical studies. Lozano et al. (2021) [27] pointed out that Ramsay scale had good application effect in the evaluation of sedation effect.

### 3.5. Incidence of Adverse Reaction

The statistical results of adverse reactions such as severe bradycardia, hypotension, hypertension, dry mouth, nausea, and vomiting in each group during the perioperative period are shown in Table 3. Through observation, the number of patients with hypotension during the perioperative period in each group was significantly higher (*P <0.05*). Okello et al. (2018) [28] raised that Dex could cause hypotension and bradycardia through pharmacodynamic analysis. Ame et al. (2020) [29] presented that hypotension was a common adverse reaction during perioperative period, which was consistent with the results of this exploration.

According to further statistics, the number of patients with adverse reactions was 12 in group A1, 12 in group A2, 7 in group A3, 18 in group B1, 19 in group B2, 18 in group B3, 17 in group C1, 15 in group C2, and 16 in group C3. It was concluded that the incidence of adverse reactions in group A3 was significantly lower than that in groups A1, A2, B1, B2, B3, C1, C2, and C3 (*P <0.05*) (Figure 9). It suggested that the incidence of adverse reactions of Dex injected at 0.8 *μ*g/(kg·h) before induction of anesthesia was better than that at 0.4 and 0.6 *μ*g/(kg·h). This was consistent with research results of *Jiang et al.* (2017) [30]. Pan *et al.* (2021) [31] presented that Dex had satisfactory sedative and analgesic effects and the incidence of adverse reactions was 0.47%.

## 4. Conclusions

It was to understand when to inject what dose of Dex for perioperative patients with the best sedative effect. In addition, many study subjects were selected nationwide, and the optimized Tri-training algorithm was adopted to classify and count the index data of the samples. The results show that NB classification algorithm has the best optimization effect; the injection of Dex at the injection rate of 0.8 *μ*g/(kg · h) before induction of anesthesia can significantly improve the fluctuation of HR, SBP, and DBP during perioperative period, and can effectively reduce the occurrence of adverse reactions in patients, which has a better sedation effect on patients. However, the formulation of Dex injection dose was not detailed enough, and there was a 0.2 *μ*g/(kg · h) difference among groups, which made the dose assessment inaccurate and needed further exploration. Nowadays, anesthesia is a necessary technique for various clinical operations, and its sedative effect has a great influence on the surgical effect and prognosis of patients. Therefore, the best application method of sedative drugs during anesthesia will be a hot topic to better benefit patients.

## Figures and Tables

**Figure 1:** Structure of Tri-training algorithm.

**Figure 2:** Optimized Tri-training algorithm process. (Training set is in the first circle, and testing set is in the second circle).

**Figure 3:** Comparison of classification effect.

**Figure 4:** Comparison of general data. (1: gynecological malignant tumor surgery; 2: laparoscopic hepatobiliary surgery; 3: subtotal thyroidectomy under general anesthesia).

**Figure 5:** Comparison of hemodynamics at 0.4 *μ*g/(kg · h). (1-before anesthesia, 2-after anesthesia, 3-during intubation, 4-5 min after intubation, 5-30 min after intubation).

**Figure 6:** Comparison of hemodynamics at 0.6 *μ*g/(kg · h). (1-before anesthesia, 2-after anesthesia, 3-during intubation, 4-5 min after intubation, 5-30 min after intubation).

**Figure 7:** Comparison of hemodynamics at 0.8 *μ*g/(kg · h). (1-before anesthesia, 2-after anesthesia, 3-during intubation, 4-5 min after intubation, 5-30 min after intubation).

**Figure 8:** Effects of different doses of Dex on HR, SBP, and DBP before induction.

**Figure 9:** Incidence of adverse reactions.

**Table 1:** Ramsay sedation scoring.

Score	1	2	3	4	5	6
Patient's condition	Not quiet irritable	Quiet cooperative	Sleepiness cooperative with doctors	Sleep state Awakenable	Not easy to wake up	Deep sleep

Note: 1--irritability; 2-4 points--satisfactory sedation effect; 5-6 points--excessive sedation.

**Table 2:** Ramsay sedation scoring of each group.

Group	Ramsay scores			Proportion of patients with satisfactory sedation effect (%)
	1	2 ~ 4	5 ~ 6	
A1 (n =55)	3	50	1	90.91
A2 (n =55)	3	49	3	89.09
A3 (n =55)	1	53	1	96.36
B1 (n =55)	4	48	3	87.27
B2 (n =55)	4	48	3	87.27
B3 (n =55)	3	50	2	90.91
C1 (n =55)	3	49	3	89.09
C2 (n =55)	2	49	4	89.09
C3 (n =55)	5	47	3	85.45

**Table 3:** Incidence of adverse reactions in each group.

Group	Adverse reactions (cases)				
	Bradycardia	Hypotension	Hypertension	Dry mouth	Nausea and vomiting
A1 (n =55)	3	11	7	2	2
A2 (n =55)	3	11	5	2	2
A3 (n =55)	1	4	2	1	0
B1 (n =55)	3	11	4	1	1
B2 (n =55)	2	13	3	2	1
B3 (n =55)	4	11	3	1	1
C1 (n =55)	4	11	2	2	1
C2 (n =55)	4	12	2	2	1
C3 (n =55)	4	13	2	1	1

## Data Availability

The datasets used and analyzed during the current study are available from the corresponding author on reasonable request.

## References

[1] Vosoughian M., Dahi M., Dabir S., Moshari M., Tabashi S., Mosavi Z. (2021). Effects of general anesthesia versus spinal anesthesia on serum cytokine release after cesarean section: a randomized clinical trial. *Anesthesiology and pain medicine*.

[2] Mei B., Li J., Zuo Z. (2021). Dexmedetomidine attenuates sepsis-associated inflammation and encephalopathy via central *α*2A adrenoceptor. *Brain, Behavior, and Immunity*.

[3] Liu X., Xie G., Zhang K. (2017). Dexmedetomidine vs propofol sedation reduces delirium in patients after cardiac surgery: a meta-analysis with trial sequential analysis of randomized controlled trials. *Journal of Critical Care*.

[4] Subramaniam B., Shankar P., Shaefi S. (2019). Effect of intravenous acetaminophen vs placebo combined with Propofol or Dexmedetomidine on postoperative delirium among older patients following cardiac surgery: the DEXACET randomized clinical trial. *JAMA*.

[5] Zeng Y., Wen Y., Yang J., Sun H. (2020). Comparing post-operative analgesic effects of varying doses of dexmedetomidine as an adjuvant to ropivacaine for ultrasound-guided dual transversus abdominis plane block following laparotomy for gynecologic malignancies. *Experimental and Therapeutic Medicine*.

[6] Naemi A. R., Kashanitabar V., Kamali A., Shiva A. (2020). Comparison of the effects of haloperidol, metoclopramide, Dexmedetomidine and ginger on postoperative nausea and vomiting after laparoscopic cholecystectomy. *Journal of Medicine and Life*.

[7] Alaa E., Adel E., Mazy A. E. (2018). Ultrasound-guided bilateral superficial cervical plexus block for thyroid surgery: the effect of dexmedetomidine addition to bupivacaine-epinephrine. *Saudi Journal of Anaesthesia*.

[8] Liu X., Song J., Zhang Y., Zhang Y., Hu X. (2021). Different Doses of Nalbuphine Combined with Dexmedetomidine in Laparoscopic Oophorocystectomy. *Medical Science Monitor: International Medical Journal of Experimental And Clinical Research*.

[9] Deiner S., Luo X., Lin H. M. (2017). Intraoperative Infusion of Dexmedetomidine for Prevention of Postoperative Delirium and Cognitive Dysfunction in Elderly Patients Undergoing Major Elective Noncardiac Surgery: A Randomized Clinical Trial. *JAMA Surgery*.

[10] Xie S., Yu Z., Lv Z. (2021). Multi-disease prediction based on deep learning: a survey. *CMES-Computer Modeling in Engineering and Sciences*.

[11] Li Y., Zhao J., Lv Z., Li J. (2021). Medical image fusion method by deep learning. *International Journal of Cognitive Computing in Engineering*.

[12] Lv Z., Qiao L. (2020). Analysis of healthcare big data. *Future Generation Computer Systems*.

[13] Chen Y., Zhou C., Li T. (2019). Named entity recognition from Chinese adverse drug event reports with lexical feature based BiLSTM-CRF and tri-training. *Journal of Biomedical Informatics*.

[14] Li Z., Togo R., Ogawa T., Haseyama M. (2020). Chronic gastritis classification using gastric X-ray images with a semi-supervised learning method based on tri-training. *Medical & Biological Engineering & Computing*.

[15] De Felice F., Crocetti D., Parisi M. (2020). Decision tree algorithm in locally advanced rectal cancer: an example of over-interpretation and misuse of a machine learning approach. *Journal of Cancer Research and Clinical Oncology*.

[16] Harada D., Asanoi H., Noto T., Takagawa J. (2021). Naive Bayes prediction of the development of cardiac events in heart failure with preserved ejection fraction in an outpatient clinic-beyond B-type natriuretic peptide. *Circulation Journal: Official Journal of the Japanese Circulation Society*.

[17] Kongsompong S., Teerasak E.-K., Chumnanpuen P. (2021). K-nearest neighbor and random Forest-based prediction of putative Tyrosinase inhibitory peptides of abalone Haliotis diversicolor. *Molecules (Basel, Switzerland)*.

[18] Shetty R. M., Bellini A., Wijayatilake D. S. (2018). BIS monitoring versus clinical assessment for sedation in mechanically ventilated adults in the intensive care unit and its impact on clinical outcomes and resource utilization. *The Cochrane Database Of Systematic Reviews*.

[19] Mansour N. A., Saleh A. I., Badawy M., Ali H. A. (2021). Accurate detection of Covid-19 patients based on feature correlated Na? Ve Bayes (FCNB) classification strategy. *Journal of Ambient Intelligence and Humanized Computing*.

[20] Wood A., Shpilrain V., Najarian K., Kahrobaei D. (2019). Private naive bayes classification of personal biomedical data: application in cancer data analysis. *Computers in Biology and Medicine*.

[21] Ngabo D., Dong W., Ibeke E., Iwendi C., Masabo E. (2021). Tackling pandemics in smart cities using machine learning architecture. *Mathematical Biosciences and Engineering: Mbe*.

[22] Ahn J. H., Kim D., Chung L. S., Lee J. J., Lee E. K., Jeong J. S. (2109). Pre-administration of remifentanil in target-controlled propofol and remifentanil anesthesia prolongs anesthesia induction in neurosurgical patients: A double-blind randomized controlled trial. *Medicine*.

[23] Li H., Liu J., Shi H. (2019). Effect of Dexmedetomidine on Perioperative Hemodynamics and Myocardial Protection in Thoracoscopic-Assisted Thoracic Surgery. *Medical Science Monitor: International Medical Journal of Experimental and Clinical Research*.

[24] Elgebaly A. S., Fathy S. M., Sallam A. A., Elbarbary Y. (2020). Cardioprotective effects of propofol-dexmedetomidine in open-heart surgery: a prospective double-blind study. *Annals of Cardiac Anaesthesia*.

[25] Shamim R., Srivastava S., Rastogi A., Kishore K., Srivastava A. (2017). Effect of two different doses of Dexmedetomidine on stress response in laparoscopic Pyeloplasty: a randomized prospective controlled study. *Anesthesia, Essays and Researches*.

[26] Ramachandran A., Palanisamy N., Vidya M. V., Zachariah M., George S. K., Ranjan R. V. (2021). Comparison of dexmedetomidine in two different doses on emergence agitation in children under sevoflurane anaesthesia: a double-blind randomised controlled trial. *Indian Journal of Anaesthesia*.

[27] Lozano-Díaz D., Valdivielso A. S., Garrido P. R., Arias‐Arias Á., Tarraga Lopez P. J., Martinez Gutierrez A. (2021). Validation of the Ramsay scale for invasive procedures under deep sedation in pediatrics. *Paediatric Anaesthesia*.

[28] Okello M. O., Mung'ayi V., Adam R., Kabugi J. (2018). A comparison of risk of hypotension using standard doses of remifentanil versus dexmedetomidine infusions in adult patients undergoing surgery under general anaesthesia at the Aga Khan University hospital, Nairobi. *African Health Sciences*.

[29] Ame A. M., Youssef A. M., El-Ozairy H. S., El-Hennawy A. M. (2020). Propofol-cetamina versus dexmedetomidina-cetamina para sedação durante endoscopia digestiva alta em pacientes pediátricos: estudo clínico randomizado. *Brazilian journal of anesthesiology (Elsevier)*.

[30] Jiang W., Wang Q., Xu M. (2017). Assessment of different loading doses of dexmedetomidine hydrochloride in preventing adverse reaction after combined spinal-epidural anesthesia. *Experimental and Therapeutic Medicine*.

[31] Pan S. Y., Liu G., Lin J. H., Jin Y. P. (2021). Efficacy and safety of Dexmedetomidine premedication in balanced anesthesia: a systematic review and meta-analysis in dogs. *Animals*.

